This article has been retracted.

# Controlled synthesis of iron oxyhydroxide (FeOOH) nanoparticles using secretory compounds from *Chlorella vulgaris* microalgae

**DOI:** 10.1080/21655979.2019.1661692

**Published:** 2019-09-09

**Authors:** Ali Ghanbariasad, Seyedeh-Masoumeh Taghizadeh, Pau Loke Show, Saifuddin Nomanbhay, Aydin Berenjian, Younes Ghasemi, Alireza Ebrahiminezhad

**Affiliations:** a Department of Medical Biotechnology, School of Medicine, and Noncommunicable Diseases Research Centre, Fasa University of Medical Sciences, Fasa, Iran; b Department of Pharmaceutical Biotechnology, School of Pharmacy, and Pharmaceutical Sciences Research Center, Shiraz University of Medical Sciences, Shiraz, Iran; c Department of Chemical and Environment Engineering, Faculty of Science and Engineering, University of Nottingham, Semenyih, Malaysia; d Institute of Sustainable Energy (ISE), Universiti Tenaga Nasional (The Energy University), Kajang, Malaysia; e Faculty of Science and Engineering, The University of Waikato, Hamilton, New Zealand; f Department of Medical Nanotechnology, School of Advanced Medical Sciences and Technologies, Shiraz University of Medical Sciences, Shiraz, Iran

**Keywords:** Carbohydrate, iron nanoparticles, iron oxide hydroxide nanoparticles, iron oxide nanoparticles, secretory compounds

## Abstract

FeOOH nanoparticles are commonly synthesized at very high temperature and pressure that makes the process energy consuming and non-economic. Recently, novel approaches were developed for the fabrication of these particles at room temperature. But, the main problem with these methods is that the prepared structures are aggregates of ultra-small nanoparticles where no intact separate nanoparticles are formed. In this study, for the first time, secretory compounds from *Chlorella vulgaris* cells were employed for the controlled synthesis of FeOOH nanoparticles at room atmosphere. Obtained particles were found to be goethite (α-FeO(OH)) crystals. Controlled synthesis of FeOOH nanoparticles resulted in uniform spherical nanoparticles ranging from 8 to 17 nm in diameter with 12.8 nm mean particle size. Fourier-transform infrared and elemental analyses were indicated that controlled synthesized nanoparticles have not functionalized with secretory compounds of *C. vulgaris,* and these compounds just played a controlling role over the synthesis reaction.

## 1. Introduction

Iron-based nanoparticles are one of the most applied nanostructures in science, technology, and medicine. These particles represent unique physicochemical and biological properties that make them interesting compounds in various fields of nanotechnology and nanosciences. Iron-based nanoparticles are now being used in diverse applications such as environmental remediation [1], microbial sciences, imaging systems [2], pharmaceutical sciences [3,4], biological products [5,6], civil engineering [7], immobilization techniques [8–10], and chemical industries [11]. Among these particles, iron oxide hydroxide (FeOOH) nanoparticles have gained unique technical applications such as pigment industries, environmental remediation, and medical supplements [12–16]. FeOOH nanoparticles have a promising capacity for toxic ion uptake and hence are widely employed in environmental remediation activities. These particles are able to remove metallic cation pollutants such as arsenic and chromium [17–19]. FeOOH nanoparticles are also able to remove fluoride from contaminated aqueous environments [20]. Besides adsorbent capacities, these particles are emerged as effective nanocatalyst in chemical reduction reactions [21].

Increasing applications of FeOOH nanoparticles in various fields resulted in increasing demand for production of these nanostructures in a sustainable manner. FeOOH nanoparticles are commonly synthesized at a high temperature which makes the process energy consuming and non-economic [22,23]. Recently, some efforts have been made to develop a procedure for fabrication of FeOOH nanoparticles at room temperature [16,24]. However, the major problem with these techniques is that the produced nanoparticles are not uniform in shape and size. For instance, Luna et al. have reported the fabrication of FeOOH nanoparticles at room temperature. The prepared particles were reported to be agglomerates of ultrafine nanoparticles with about 3.3 nm in diameter. The authors also reported the presence of some large rod-like structures with 23 ± 5 nm in length and 5 ± 1 nm in width [24]. Similar problems were found in the biosynthesized nanoparticles using *Klebsiella oxytoca* and *Ralstonia* sp. [25,26].

Previous investigations revealed that both intracellular and extracellular bioactive compounds from *Chlorella vulgaris* microalgae can play a shape-directing role in the fabrication of metallic nanoparticles [27–29]. Algal proteins and carbohydrates were identified as the main intracellular and secretory shape-controlling factors, respectively [27–29]. The carboxyl groups in Asp and/or Glu residues of algal proteins were driving the anisotropic growth of Ag nanocrystals into nanoplates [28,29]. Nevertheless, secretory carbohydrates made the particles fairly uniform in both shape and size. Also, secretory carbohydrates controlled the nanoparticle growth pattern and induced isotropic growth of nanocrystals [27]. The present investigation, therefore, aims at evaluating secretory carbohydrates from *C. vulgaris* for shape-controlling fabrication of uniform FeOOH nanoparticles at room atmosphere.

## 2. Materials and methods

### 2.1. Materials

All chemicals were purchased from Merck in analytical grade and used as received without any further purification. Millipore water (resistance >18 MΩ cm^−1^) was used throughout the experiment.

### 2.2. Culture of microalgal cells

*C. vulgaris* cells were cultured (10^7^ cell ml^−1^) in 250 ml Erlenmeyer flask containing 100 ml of BG-11 broth medium and incubated at 27°C in 16 h light/8 h dark cycle with light intensity of 60 μ Em^−1^ s^−1^ cool white fluorescent lamp. After 20 days, at the end of growth logarithmic phase, cells were harvested by centrifugation, and the supernatant was employed for nanoparticle synthesis [27].

### 2.3. Uncontrolled synthesis of FeOOH nanoparticles

Uncontrolled synthesis of FeOOH nanoparticles was performed as described previously by Luna et al. with some modification [24]. Briefly, 1.1 g FeCl_3_.6H_2_O was dissolved in 25 ml deionized water and then 30 ml sodium hydroxide solution (5 M) was rapidly added to start the reaction. The mixture was maintained 15 min under vigorous steering at room atmosphere. The resulting suspension was centrifuged at 4000 rpm for 20 min. The precipitate was washed three times by deionized water and dried in an oven at 50°C for 48 h.

### 2.4. Controlled synthesis of FeOOH nanoparticles

Controlled synthesis of FeOOH nanoparticles was performed in the presence of *C. vulgaris* secretory carbohydrates. Briefly, 1.1 g FeCl_3_.6H_2_O was dissolved in 25 ml culture supernatant and then 30 ml sodium hydroxide solution (5 M) was rapidly added under vigorous steering. The reaction was followed for 15 min at room temperature. The dark brown precipitate was harvested by centrifugation at 4000 rpm for 20 min. The resulting precipitate was washed three times by deionized water and dried in an oven at 50°C for 48 h.

### 2.5 Characterization of the synthesized nanoparticles

A drop of the prepared nanoparticle suspension was dripped on a carbon-coated grid Cu Mesh 300 Formvar and dried at room temperature. Transmission electron microscopy (TEM) analysis was done by using Zeiss EM10C, TEM, operated at HT 80 kV. Diameters of 100 particles were measured randomly using ImageJ (version 1.47v), an image analyzing software developed by the National Institutes of Health (http://imagejnihgov/ij/). Fourier-transform infrared (FTIR) spectroscopy analysis was done on a PerkinElmer FTIR spectrometer using KBr pellets. The crystallinity of the particles was evaluated by x-ray diffraction patterns (XRD, Siemens D5000) using fine powder of nanoparticles. Chemical composition of the sample was analyzed by using a CHNS elemental analyzer (Costech, ECS 4010).

## 3. Results and discussion

By the addition of sodium hydroxide solution to the reaction mixture, a sudden change in the color was occurred from light orange to yellowish-brown, suggesting the formation of iron oxyhydroxide (FeOOH) colloidal suspension. In this reaction, FeOOH nanoparticles precipitate upon hydrolysis of ferric ions. Sodium hydroxide acts as a precipitating agent and FeOOH nanoparticles are formed as represented in Equation (1) [12,30].

(1) $$Fe^{3+}\;+3OH^{-}\;\to \;Fe{\left(OH\right)}_{3}\;\to \;FeOOH+H_{2}O$$

After centrifugation and harvesting FeOOH nanoparticles, a completely clear supernatant was obtained. TEM micrographs revealed that uncontrolled synthesis of FeOOH nanoparticles resulted in large aggregates of ultrafine nanoparticles (Figure 1(a)). However, controlled synthesis in the presence of secretory carbohydrates from *C. vulgaris* resulted in the discrete spherical nanoparticles ranging from 8 to 17 nm in diameter with an average size of 12.8 nm (Figures 1(b) and 2). It has been reported that uncontrolled synthesis of FeOOH nanoparticles at room temperature resulted in the aggregates of ultrafine nanoparticles. At this reaction condition also, a second community of large nanorods can be observed [24]. In this experiment, the presence of secretory carbohydrates in the controlled synthesis reaction inhibited the formation of second community of large nanostructures. These results are in close agreement with previous findings of the shape-controlling effect of the secretory carbohydrates from *C. vulgaris* [27]. In addition, a similar controlling effect was reported for monosaccharides such as dextrose [31]. It is believed that carbohydrates can control the reaction in both nucleation and growth phases. In the nucleation phase, carbohydrates prevent monotonic nucleation by chelation of iron ions and limit the size of nuclei. In the growth phase, carbohydrates control the growth of formed nuclei and inhibit the formation of large particles [31]. Besides biochemical species, chemical polymers can also control the fabrication of FeOOH nanoparticles and are employed for the shape- and size-controlled synthesis reactions [32]. It is obvious that reaction protocol and reaction conditions are other parameters that can control the resulted particle size and morphology [33,34].

**Figure 1.** TEM micrographs of the uncontrolled (a) and controlled (b) synthesized FeOOH nanoparticles.

**Figure 2.** Particle size distribution of the controlled synthesized FeOOH nanoparticles.

FTIR spectra of uncontrolled and controlled synthesized particles were recorded and depicted in Figure 3. Characteristic peak of iron oxides which is from Fe–O bond was appeared at 617 cm^−1^ [5,35,36]. The peak at 1339 cm^−1^ is usually considered as C–O groups which may be from impurities. The O–H groups deforming and stretching vibration recorded at about 1502 and 3360 cm^−1^, respectively. It has been reported that polysaccharides like guar gum and xanthan gum could be adsorbed to the surface of iron-based nanoparticles [1]. Also, it has been shown that secretory carbohydrates from *C. vulgaris* can engulf silver nanoparticles in about 1 nm thickness. However, in the case of controlled synthesized FeOOH nanoparticles, secretory carbohydrates from *C. vulgaris* have not played any capping role.

**Figure 3.** FTIR spectra of the uncontrolled (a) and controlled (b) synthesized FeOOH nanoparticles.

XRD patterns of the uncontrolled and controlled synthesized nanostructures are shown in Figure 4. Recorded spectra revealed that the prepared structures are nanocrystals of goethite (α-FeOOH) [37]. The similarity in the crystalline structure of the uncontrolled and controlled synthesized nanoparticles revealed that secretory carbohydrates from *C. vulgaris* have not disturbed or modified the formation of nanocrystals. The recorded patterns seem to be nearly amorphous. However, similar broad hump-like peaks with very low intensity are usual for FeOOH nanoparticles [38]. Based on the pattern, both uncontrolled and controlled synthesized nanoparticles can be assigned to goethite (α-FeOOH) (JCPDS No. 22-0713) [32,39,40].

**Figure 4.** XRD pattern of the uncontrolled (a) and controlled (b) synthesized FeOOH nanoparticles. (c) XRD pattern of goethite crystals based on JCPDS card No. 22-0713.

Results for elemental analysis of the prepared nanostructure are tabulated in Table 1. The corresponding CHNS chromatogram is also shown in Figure 5. Nitrogen, carbon, and hydrogen are made 0.02, 1.56, and 0.91 weight percent of the uncontrolled synthesized nanomaterial, respectively. These data are not significantly different from the uncontrolled synthesized nanoparticles. Elemental content of the controlled synthesized nanostructures was measured as N/A, 0.59, and 1.03 for nitrogen, carbon, and hydrogen, respectively. These data are supporting the FTIR findings and confirm that secretory carbohydrates from *C. vulgaris* have a capping role in the formation of controlled synthesized FeOOH nanostructures. In addition to the previous report which has been shown that secretory carbohydrates from *C. vulgaris* can play a capping role in biologically synthesized silver nanoparticles [27], similar results were also reported for biosynthesized FeOOH nanoparticles. Carbohydrate contents of the biosynthesized nanoparticles were reported to be 17 and 25 weight percent in the case of *K. oxytoca* and *Ralstonia* sp. synthesized nanoparticles, respectively [25,26]. Preparation of pure FeOOH nanoparticles without the addition of any biological compound or surface modification can be a significant advantage as these particles are suitable for any required functionalization.

**Figure 5.** CHNS chromatogram of the uncontrolled (a) and controlled (b) synthesized nanoparticles.

**Table 1.** Elemental composition (nitrogen, carbon, and hydrogen content) of the prepared nanostructures recorded by a CHNS elemental analyzer.

Element	Retention time (min)		Weight (mg)		Weight (%)	
Sample	Uncontrolled synthesized	Controlled synthesized	Uncontrolled synthesized	Controlled synthesized	Uncontrolled synthesized	Controlled synthesized
N	1.257	1.287	0.001	N/A	0.02	N/A
C	2.517	2.520	0.062	0.018	1.56	0.59
H	8.207	8.073	0.036	0.032	0.91	1.03
Total	-	-	3.993	3.071	2.49	1.62

## 4. Conclusions

Culture supernatant of *C. vulgaris* is abundant with bioactive compounds where carbohydrates are the major part of these biomolecules. Current investigation revealed that culture supernatant of the *C. vulgaris* can be employed as a sustainable source of bioactive compounds for the controlled synthesis of FeOOH nanoparticles at ambient atmosphere. The prepared particles were pure (free of any biologic compound), spherical, uniform, and in the size range that is ideal for nanostructures. Characteristic advantages of the controlled synthesized nanoparticles over uncontrolled synthesized FeOOH can make them a promising substitute for previously employed particles.

## Highlights

- FeOOH nanoparticles were fabricated in a controlled synthesis reaction.
- Secretory compounds from *C. vulgaris* were used as a controlling agent.
- Secretory compounds have not disturbed or modified the formation of nanocrystals.
- Small nanospheres with a narrow particle size distribution were resulted.
- The resulted structures were uniform in shape and size.
